RETRACTED

# Impact of Cluster Nursing on Nursing on VAS Score and Urinary Function of Patients after Percutaneous Nephrolithotomy with Pneumatic Lithotripsy (PCNL)

**DOI:** 10.1155/2022/3743640

**Published:** 2022-03-19

**Authors:** Zhengyuan Li, Hong Chen, Shiduo Zhao, Gangtian Yang, Wenfan Yang, Jingping Guo

**Affiliations:** Urology Surgery, The First Affiliated Hospital of Kangda College of Nanjing Medical University (The First People's Hospital of Lianyungang), Lianyungang 222061, China

## Abstract

**Objective:**

To explore the effects of cluster nursing on VAS score and urinary system function of patients after percutaneous nephrolithotomy with pneumatic lithotripsy (PCNL).

**Methods:**

November 2019-January 2019, 114 patients with PCNL who received treatment in our hospital were selected and randomly divided into two groups: the control group and the study group. The study group received cluster nursing, and the control group received routine nursing. Compare the Barthel index (BI), between two groups, SAS score, complications rate, surgical outcomes, pain scores, quality of life scores, knowledge awareness rate, and satisfaction rate were compared.

**Results:**

There were no significant variations in Bi and SAS scores before the nursing (*P* > 0.05). The BI ratings were clearly higher after nursing, whereas the SAS and pain levels were considerably lower, however, the research group altered more dramatically (*P*0.05). The study group's incidence of complications was lower (*P*0.05) than the control group's; the study group's hospitalization cost was lower, and the hospitalization and lower bed activity were shorter (*P*0.05); after the nursing, the organised quality score was significantly higher in both groups, but the research group changed more dramatically (*P*0.05). Compared with the control group, the knowledge of the research team was higher (*P* < 0.05); after the nursing, both group satisfaction scores were obviously high, but the study group changes more significantly (*P* < 0.05).

**Conclusion:**

After PCNL treatment, the patient receives cluster therapy, improving the patient's anxiety, reducing the degree of pain, and improving the quality of life in patients, and the patient satisfaction is high. Therefore, cluster nursing is worthy of extensive application in the postoperative care of patients with PCNL.

## 1. Introduction

Kidney stones are obviously repeatable characteristic disease, a higher incidence of high urinary diseases, and are more harmful. In particular, multiple kidney stones, if there is no timely effective treatment, it will damage the kidney function, increase the incidence of uremia [1]. Long-term, food structure, and drinking water are the ones that are less affected by the sickness. The present medical level has advanced at a quick pace. The proliferation of lens and kidney mirror is more widespread in clinical therapy. This therapy may be removed successfully, which leads to an improvement in clinical symptoms, a quick postoperative recovery, and little stress and blood loss. Less, etc., results in greater therapeutic efficacy and safety and is the initial treatment approach [2, 3]. Nonetheless, intraoperative disinfection, infusion temperature, anaesthesia method, skin exposure, and other factors can influence the treatment process, resulting in lower body temperatures in patients, which increases the risk of surgery, and postoperative patients will experience varying degrees of pain and complications, as well as depression and anxiety [4]. As a result, multidimensional nursing should be provided. Cluster nursing for patients following PCNL surgery may achieve psychological and complications nursing, with perfect nursing effect and a significant role in improving patient prognosis, according to this research [5, 6].

RETRACTED

The study chose 114 patients with PCNL treatment in our hospital, analyzing the impact of packed VAS scores after PCNL, as reported below.

## 2. Data and Methods

### 2.1. General Information

A total of 114 patients receiving PCNL treatment in our hospital from January 2019 to January 2021 were selected. The control group (*n* = 55) consisted of 28 males and 27 females, aged 18-71 years, with an average age of (45.3 ± 5.1) years, with a disease course of 1-6 years and an average disease course of (3.1 ± 0.6) years. There were 11 cases of right kidney stone, 12 cases of left kidney stone, and 32 cases of double kidney stone. In the study group (*n* = 59), there were 30 males and 29 females, aged 18-71 years, with an average age of (45.1 ± 4.8) years, with a disease course of 1-6 years, with an average of (2.9 ± 0.5) years, and 55 patients, including 12 cases of right kidney stone, 14 cases of left kidney stone, and 33 cases of double kidney stone, respectively. The research object agreed that the information was comparable (*P* > 0.05) and was approved by the Hospital Ethics Committee.

Inclusion criteria [7]: (1) persons aged 18 to 80; (2) PCNL indications; (3) kidney stones confirmed by pathology, abdomen CT, or intravenous urography; (4) those who are aware of the research and have signed the informed agreement; (5) heart rate and blood pressure were steady and satisfactory.

Excluding criteria: (1) language or consciousness; (2) kidney, cardiopulmonary disease; (3) acute and chronic infection; (4) urinary tract deformity; (5) malignant tumor; (6) chronic pain disease; (7) cardiovascular and cerebrovascular diseases.

RETRACTED

## 3. Method

Regular care: preoperative heart rate, blood pressure, and other routine examination of patients, and to tell patients about the disease and surgical treatment related knowledge, with psychological intervention. Assist the operation after operation, transfer surgical instruments to the operator in time. Postoperative attention to the patient should be explained.

Cluster nursing: (1) the head of the nurse serves as the team leader, and the team members include the nurse, the nurse, and the responsible nurse. The use of slideshows to teach complications and trigger problems together taught complications and provoked complications. The members of the team must gather relevant research on perioperative problems, synthesise it, and then coordinate nursing interventions. (2) Surgical procedures: 1 hour before operation, check that the control room temperature is 25°C by preheating the operating room. During the transfer, the patient will be kept warm with a quilt and blanket cover. The lavage and infusion fluids should be heated to 37°C intraoperatively. Purulence secretions surrounding the fistula mouth were studied, urine characteristics and color were noted, and the fistula was appropriately fastened to prevent the pipeline sliding or tugging. If there is a pattern of extrusion or pipe clogging, the drainage tube should be washed on a regular basis. Furthermore, the fistula must be sterilised, and the skin must be maintained dry and clean. (3) Pain care: the patient will be accompanied by different degrees of pain, including the skin pain around the fistula, interpret the patient to the patient, and give Lendocaine for local analgesic pain. Nursing staff should regularly participate in intellectual lectures, learn to nursing skills and pain knowledge, formulate workflows, and standardize management. It is given sedation or analgesic treatment based on the patient's specific situation. (4) Complications care: observe the drainage, drainage color, and vital signs, if there is a large amount of fresh red blood liquid in a short time, the patient is accompanied by pulse and blood pressure reduction, the drainage tube should be closed immediately, and this is immediately informed to the Doctor. After surgery, clean the urine port and pine promptly, change the fistula dressing on a regular basis, and maintain the skin dry and clean. If the patient has nephrosis, the fistula is utilised to rinse with physiological saline, and the fistula's distal end is extruded. (5) Psychological care: patients who do not comprehend the concepts of therapy are concerned about the prognosis and are depressed or anxious will have a significant impact on treatment outcomes. Nursing workers should provide information and instruction to patients, as well as care and encouragement, in order to increase favourable treatment outcomes.

RETRACTED

### 3.1. Observation Indicator

Barthel index (BI) [8]: the patients' acceptance ability, indwelling catheter, state of consciousness, active nutrition, physical tolerance, vital signs, emotional state, renal fistula drainage, and stoma were analyzed. The total score was 100, and the higher the score, the better the life ability. *Anxiety (SAS) Rating* [9]. Evaluation of patient anxiety, a total of 20 projects, 50 are divided into standard points, patient anxiety degree is negatively correlated with the standard points. *Complications Incidence*. Statistical infection, urinary fistula, number of bleeding, and calculation rate. *Surgical Results*. Including hospitalization costs, hospitalization, and the activity time of ambulation of approximately 10 cm. *Pain Rating*. Applying about 10 cm long swatches to the patient's pain level, 0-10 scale corresponds to 0-10 points, patients evaluate the degree of pain in their own pain, and patient pain levels are positively correlated with the score. *Life Quality Rating* [10]. Social function, physiological functions, mental health, physical pain, emotional function, etc. Evaluation, total 100 points, patient satisfaction, and score positively correlation. *Satisfaction Rating* [11]. Applying the satisfaction survey of the court to the patient satisfaction evaluation, including nursing technology, protective communication, health education, and ward environment. The total is 100 points, and the score is greater than 80 points.

### 3.2. Statistical Method

Data application statistics SPSS22.0 software analysis, for statistical analysis of the Zhengtai distribution data, the measurement data is expressed, and the difference between two groups is selected, enter the acquired data into the Excel form, data application statistics SPSS22.0 software analysis, for statistical analysis of the Zhengtai distribution data, the measurement data is expressed, and the difference between two groups is selected. The count data is stated (for example, in percent), and the physical impact factor of the case group is used to pick the card-calibration component differential data. The research institution is employed as the picture software for graphpad prism, which uses logistic regression analysis and *P*0.05 as the statistical significance.

## 4. Results

Bi, SAS score compared before care, Bi, SAS scores have no significant difference in both groups (*P* > 0.05), after nursing, the BI scores increase significantly, SAS scores are significantly reduced, but the research group changes more clearly. There is a statistical significance of intergroup comparison (*P* < 0.05), shown in Table 1.

RETRACTED

Comparison of incidence of complications in two groups compared to the comparison group, the incidence of complications in the study group is 10.9%, 5.1%, respectively, compared with the control group, the incidence of complications of the study group is lower, compared between groups, and statistical significance (*P* < 0.05), shown in Table 2.

Comparison of surgery results in two groups Compared to the control group, the research team was lower, and the hospitalization and the lower bed activity were shorter (*P* < 0.05) (Table 3).

Comparison of pain scores. After two treatments, two groups were significantly lower pain scores, the study group but decreased pain scores more significant, comparisons between groups, statistically significant difference (*P* < 0.05), shown in Figure 1.

Comparison of quality of life score in two groups. Before treatment, there was no significant difference in quality of life scores between the two groups (*P* > 0.05), but after treatment, both groups had significantly higher quality of life scores, with more significant changes in the study group, compared between groups, statistically significant differences (*P*0.05), as shown in Figure 2.

Comparison of knowledge rate in two groups. Knowledge rate was 86.3% and 96.6%, respectively, in two groups, and awareness rate of study group is higher (*P* < 0.05), shown in Figure 3.

Comparison of satisfaction scores in two groups. Compared to the previous two treatments, two satisfaction scores were not significantly different (*P* > 0.05); after treatment, satisfaction scores were significantly higher in both groups, but more significant changes in the study group. And compared between two groups, differences were statistically significant (*P* < 0.05), shown in Figure 4.

## 5. Discussion

Percutaneous nephrolithotomy pneumatic lithotripsy in the treatment of kidney stone lithotripsy has improved in recent years due to the fast development of minimally invasive medicine [12, 13]. However, many elements may influence therapy; patients may experience hypothermia, which reduces the body's immune system and affects coagulation; thus, in order to increase treatment safety, acceptable intervention should be compatible [14].

Nurses may enhance the quality of care by clustering care and providing frequent training to nurses in order to actively anticipate issues that may arise during care [15]. It is crucial that we can engage via appropriate treatments to lower the occurrence of adverse events [16]. The findings revealed that the incidence of complications in the study group was 10.9 percent, 5.1 percent lower than the control group study group complication rate. The findings revealed that cluster nursing can enhance patient outcomes by reducing the prevalence of urinary fistula complications such as bleeding and favouring infection. Postoperative patients in various levels of pain would, to a significant extent, alter the patients' excitement [17]. As a result, postoperative pain requires nursing involvement; nurses must measure the degree of pain in patients, and sedative and analgesic therapy may successfully decrease pain in patients, as well as the accompanying negative emotions [18, 19]. The study results show that the impact of cluster analysis study of patient care VAS score after PCNL, study results showed that after treatment, the two groups BI scores were significantly increased, SAS and pain were significantly reduced, but the changes are more obvious in research group (*P* < 0.05), and the result of research and clinical findings of other scholars has higher consistency [20], and thus show that the cluster of nursing intervention should be widely applied. In the study, knowledge awareness and satisfaction change were investigated after patients were bundled nursing intervention, patients received health education, prevention, and intervention through reasonable measures, and it can improve the degree of cognitive disorders in patients [21–23]. The results showed that the study group's knowledge rate was 86.3 percent, and the control group was 96.6 percent, respectively, and that the study group's awareness of knowledge was higher (*P*0.05) than the control group. After treatment, both groups had significantly higher satisfaction scores, but the study group had more significant changes (*P*0.05). This finding demonstrates that a large cluster of care apps may enhance clinical outcomes in patients and provide complete care. Current clinical nursing care, guided by the “patient-centered” philosophy, is concerned not only with the patient's physical recovery but also with his or her emotional and psychological well-being, with the intention of improving the patient's functions by active intervention [24–26]. The study patients after PCNL cluster of nursing care can be an effective combination of caring elements, a relatively routine care can improve the quality of life to a greater extent, and high patient satisfaction degree.

RETRACTED

In summary, cluster nursing treatment for PCNL patients after treatment can improve patients' anxiety, reduce the degree of pain, and improve the quality of life of patients, patients with high satisfaction. Therefore, cluster nursing is worthy of extensive application in the postoperative care of patients with PCNL.

## Figures and Tables

**Figure 1:** Comparison of pain scores.

**Figure 2:** Comparison of quality of life score in two groups.

**Figure 3:** Comparison of knowledge rate in two groups.

**Figure 4:** Comparison of satisfaction scores in two groups.

**Table 1:** Comparison of BI and SAS scores between the two groups ().

Group	Count	BI rating (minute)			SAS score (minute)		
		Before the care	7 days after the care	14 days after care	Before the care	7 days after the care	14 days after care
Control group	55	62.9 ± 5.2	66.7 ± 5.9	70.5 ± 7.1	44.2 ± 5.1	41.9 ± 4.3	39.6 ± 3.7
Research group	59	62.7 ± 5.1	76.8 ± 6.2	84.6 ± 7.5	44.1 ± 4.8	37.1 ± 3.8	32.2 ± 3.5
*T*	/	0.527	16.482	17.024	1.862	14.028	13.759
*P*	/	>0.05	<0.05	<0.05	>0.05	<0.05	<0.05

**Table 2:** Comparison of incidence of complications in two groups (example, %).

Group	Count	Infect	Urinary fistula	Bleeding	Incidence
Control group	55	2(3.6)	3(5.5)	1(1.8)	10.9%
Research group	59	1(1.7)	2(3.4)	0(0.0)	5.1%
*X* ^2^	/	/	/	/	6.018
*P*	/	/	/	/	<0.05

**Table 3:** Comparison of surgery results in two groups ().

Group	Count	Hospitalization costs (million yuan)	Length of stay (d)	Ambulation (d)
Control group	55	1.7 ± 0.5	13.4 ± 2.5	5.3 ± 1.2
Research group	59	1.2 ± 0.4	9.6 ± 1.4	3.1 ± 0.8
*X* ^2^	/	13.724	15.631	14.524
*P*	/	<0.05	<0.05	<0.05

## Data Availability

The data used to support the findings of this study are included within the article.
